The article "Sec-O-glucosylhamaudol suppressed inflammatory reaction induced by LPS in RAW264.7 cells through inhibition of NF-κB and MAPKs signaling" was published in 2020. Journal: Biosci Rep.

# Sec-O-glucosylhamaudol suppressed inflammatory reaction induced by LPS in RAW264.7 cells through inhibition of NF-κB and MAPKs signaling

**DOI:** 10.1042/BSR20194230

**Published:** 2020-02-14

**Authors:** Guiming Liu, Jing Xie, Yurui Shi, Rongda Chen, Li Li, Mengxue Wang, Meizhu Zheng, Jiaming Xu

**Affiliations:** 1 The College of Chemistry, Changchun Normal University, Changchun 130032, China; 2 The College of ChangChun University of Chinese Medicine, Changchun 130036, China

**Keywords:** inflammation, LPS, macrophages, MAPKs, NF-κB, SOG

## Abstract

As a major bioactive compound from the *Saposhnikovia divaricata (Turcz.) Schischk*, sec-O-glucosylhamaudol (SOG), has been reported to have anti-nociceptive activity and high 5-lipoxygenase (5-LOX) activity. Nevertheless, the mechanism of the potential anti-inflammatory effects of SOG is unclear. The anti-inflammatory impacts of SOG in RAW 264.7 cell lines stimulated by LPS were explored in the present study. It was found that SOG dose-dependently reduced the emergence of inflammation cytokines, such as IL-6 and TNF-α in Raw264.7 murine macrophages stimulated by LPS. Real-time PCR assay demonstrated the SOG dose-dependently inhibited transcription of these cytokines as well. In addition, it was also found that NF-κB activation and MAPKs phosphorylation including p38, JNK and ERK1/2 induced by LPS were suppressed by SOG. Due to its anti-inflammatory activity, our results suggest that SOG might have therapeutic effects on inflammatory disease, such as acute lung injury or rheumatoid arthritis.

## Introduction

Inflammation is considered to be a complicated biological process in which a host identifies substances in or out of the body as self-antigens or non self-antigens. A proper inflammatory reaction helps the host to resist the invasion of pathogens, while uncontrolled inflammation will cause massive tissue injury, thus showing pathological condition. Some studies have shown that activated macrophages are the main pro-inflammatory cells, which mediate most cellular and molecular inflammatory networks via releasing a variety of inflammatory mediators [1].

Lipopolysaccharide (LPS) is an important component of Gram-negative bacteria’s outer membrane. After interaction with CD14, Toll-like receptor 4 and MD-2 on the cell surface, LPS can stimulate macrophages to produce inflammatory mediators including TNF-α, ILs, iNOS and COX-2 [2,3]. Meanwhile, the IкB kinase (IKK)-NF-кB and three mitogen-activated protein kinase (MAPK) pathways were also activated by these interactions [4].

As a traditional Chinese medicine, *Saposhnikovia divaricata* (Turcz.) Schischk has been reported to treat headache, generalized aches, inflammation and cancer in China [5,6]. SOG is a major bioactive compound from *S. divaricata* [7], which has been reported to have antinociceptive activity [8]. Even more, it is an important component of a famous Chinese medicine Yupingfeng [9]. In our previous study, SOG showed a high inhibition of 5-LOX activity with an IC_50_ of 7.45 µM *in vitro* [10]. Nevertheless, whether and how SOG exerts anti-inflammatory effects remain unclear. Therefore, whether SOG inhibits Raw264.7 macrophages activation induced by LPS and its anti-inflammatory mechanism is elucidated in the present study.

The article "Sec-O-glucosylhamaudol suppressed inflammatory reaction induced by LPS in RAW264.7 cells through inhibition of NF-κB and MAPKs signaling" was published in 2020. Journal: Biosci Rep.

## Materials and methods

### Chemicals and reagents

SOG was bought from Shanghai Yuanye Bio-Technology (Shanghai, China). RPMI 1640 Medium, TRIzol reagent, fetal bovine serum (FBS), streptomycin and penicillin were from Invitrogen-Gibco (Grand Island, NY, U.S.A.). LPS, dimethyl sulfoxide (DMSO) and 3-(4,5-dimethylthiazol-2-yl)-2,5-diphenyl tetra-zolium bromide (MTT) were obtained from Sigma-Aldrich (St. Louis, MO, U.S.A.). Enzyme-linked immunosorbent assay (ELISA) kits for IL-6 and mouse TNF-α were obtained from eBioscience (San Diego, CA, U.S.A.). The antibodies against phosphorylated proteins including p65, ERK1/2, p38, JNK and β-actin were obtained from Cell Signaling Technology (Danvers, MA, U.S.A.). Other antibodies applied in the present study were from Bioworld (St. Louis Park, MN, U.S.A.).

### Cell culture and MTT assay

RAW264.7 cells were cultured in RPMI 1640 medium, which is added with 10% heat-inactivated FBS and 1% penicillin–streptomycin solution (complete medium), cells were then placed in a humidifying incubator in the environment filled with 5% CO_2_ at 37°C. Cells were seeded in 96-well plates at 5 × 10^4^ cells/well, which was then cultured with complete RPMI 1640 medium over one night. Treated with or without LPS (500 ng/ml), cells were incubated with three doses of SOG (25, 50, 100 μM) for 24 h. According to the manufacturer’s protocol, MTT assays were then performed. Briefly, after washing twice with PBS, cells were incubated in complete medium added with 0.5 mg/ml MTT filled with 5% of CO_2_ at 37°C. Four hours later, the medium was aspirated, and the reduced product of MTT, formazan, was dissolved in DMSO. Then, a microplate reader was applied to measure the optical density at 490 nm. RAW264.7 cell viability was expressed as a percentage of untreated control group.

### Detection of cytokines by ELISA analysis

RAW264.7 cells were seeded in 24 well plates with 2 × 10^5^ cells/well, then incubated overnight in RPMI 1640 complete medium in a humidified incubator filled with 5% CO_2_ at 37°C overnight. After changing medium, cells were processed with 500 ng/ml LPS and indicated three concentrations of SOG at 25, 50, 100 μM for 6 h, and culture supernatants were collected and frozen for ELISA assay at −80°C. According to the instruction of producers, the cytokines released into the culture supernatant were measured by ELISA assay as described previously [11]. In short, the ELISA plate was coated with primary antibody and diluted with carbonate–hydrocarbonate buffer at 4°C overnight. After cleaning three times with PBS, the samples were put into duplicate wells, and the plates were incubated for 2 h at 37°C. After washing three times with PBS, biotin-conjugated polyclonal antibody was put to each well, and incubated for 2 h at 37°C. After washing three times with PBS, streptavidin HRP was put to each well. The plates were washed completely for five times, and TMB substrate was added after incubation for 1 h. Terminating buffer was finally added to stop reaction after 0.5 h at room temperature. A microplate reader was applied to measure the optical density at 450 nm.

The article "Sec-O-glucosylhamaudol suppressed inflammatory reaction induced by LPS in RAW264.7 cells through inhibition of NF-κB and MAPKs signaling" was published in 2020. Journal: Biosci Rep.

### RNA extractions and qPCR analysis

RAW264.7 cells were seeded in plates with six cells at 1 × 10^6^ cells/well in RPMI 1640 complete medium, and cultured overnight in a humidified incubator with 5% CO_2_ at 37°C. Cells were then treated with 500 ng/ml LPS and indicated three concentrations of SOG (25, 50, 100 μM) for 1 or 6 h. After removing media, 300 μl TRIzol reagent was added to each well to lyse cells. The extraction of RNA was conducted on the basis of the instructions of producers, along with the transcription of RNA samples into cDNA employing Transcriptor First Strand cDNA Synthesis Kit (Roche, Basel, Germany). In ABI 7500 real-time PCR system (Applied Biosystems, Carlsbad, CA), SYBR Green PCR master mix reagent kit (Takara, Dalian, China) was used to measure the mRNA level of the selected gene. The primers used for PCR are as follows: TNF-α: 5′-GGCTCCAGGCGGTGCTTGTT-3′ and 5′-GGCTTGTCACTCGGGGTTCG-3′; IL-6: 5′-GGATACCACTCCCAACAGACC-3′ and 5′-TCCAGTTTGGTAGCAT CATCA-3′; β-actin: 5′-GATCAAGATCATTGCTCCTCCTG-3′ and 5′-AGGGTGTAAAACGCAGCTC. The calculation of relative quantity of genetic expression was achieved on the basis of the formula below: 2^−△△*C*t^, where △*C*t = [*C*t (gene) *C*t (β-actin)] and *C*t is the crossing threshold value of each gene amplification returned by the PCR.

### Western blot assay

RAW264.7 cells were seeded in dishes with 6 cm at 2 × 10^6^ cells/well in RPMI 1640 complete medium in a humidifying incubator filled with 5% CO_2_ at 37°C overnight. Cells were processed with 500 ng/ml LPS, and indicated three concentration of SOG (25, 50, 100 μM) after changing of medium. After washing three times with ice-cold PBS, cells were lysed in RIPA buffer consisted of 150 mM NaCl, 50 mM Tris, pH 7.4, 1% NP-40, 0.5% sodium deoxycholate and 0.1% SDS. The supernatant was collected after being centrifuged at 14,500 ***g*** at 4°C for 20 min. A BCA-protein assay kit (Wanleibio, Shenyang, China) was employed to determine contents of protein of samples. Fifty micrograms of protein were isolated using 12% SDS-PAGE and electro-transferred to a PVDF membranes (Millipore, U.S.A.). The membranes were blocked by TBST containing 3% BSA for 2 h at room temperature, and probed with various primary antibodies at 4°C overnight. After being washed three times with TBST at intervals of 10 min, membranes were incubated with horseradish peroxidase-conjugated secondary antibodies for 1 h at room temperature. After three times of washing, the immunoreactive bands were visualized using chemiluminescent substrate of SuperSignal West Pico (Thermo, U.S.A.) and were further quantified using ImageJ software (National Institutes of Health, U.S.A.).

The article "Sec-O-glucosylhamaudol suppressed inflammatory reaction induced by LPS in RAW264.7 cells through inhibition of NF-κB and MAPKs signaling" was published in 2020. Journal: Biosci Rep.

### Data analysis

Experimental data were expressed by mean ± SD. Using GraphPad Prism 4.0 software (GraphPad Software, Inc., San Diego, CA) to analyze differences among the various treatment groups by one-way analysis of variance (ANOVA). The difference was statistically significant at *P* < 0.05, and the difference was extremely significant at *P* < 0.01 or *P* < 0.001.

## Results

### SOG suppressed inflammatory cytokines release in LPS-stimulated macrophages

To investigate whether SOG possessed anti-inflammatory activity, the effect of SOG on production of TNF-α and IL-6 in LPS-stimulated RAW264.7 murine macrophage cells were examined. As shown in Figure 1, the contents of TNF- α and IL-6 in the supernatant of LPS-treated cells were compared with those of untreated cells. As a result, SOG treatment markedly decreased the emergence of these inflammatory cytokines stimulated by LPS in a dose-dependent manner.

**Figure 1:** SOG inhibits the release of inflammatory cytokines Indicated concentrations of SOG (25, 50 and 100 μM) were added to RAW 264.7 cells stimulated by LPS. Supernatant medium was collected after 6 h of incubation, and TNF-α (**A**) and IL-6 (**B**) were detected by ELISA. The results of three independent experiments were expressed as means ± SEM. ^###^*P* < 0.001 versus blank group (LPS-unstimulated cells), *P < 0.05, **P < 0.01 and ***P < 0.001 versus group treated by LPS.

### Effects of SOG on the viability of LPS-stimulated macrophages

In order to eliminate the possibility that the cytotoxic effect of SOG can inhibit the production of inflammatory cytokines stimulated by LPS, the potential cytotoxicity of SOG at 25, 50, 100 μM was further assessed by MTT method after 24 h of culture with LPS. As shown in Figure 2, SOG showed no significant cytotoxicity when the concentration reaches 100 μ M, indicating that the inhibitory effect of SOG on LPS-induced TNF- α and IL-6 was not affected by the potential cytotoxic effect of this compound.

The article "Sec-O-glucosylhamaudol suppressed inflammatory reaction induced by LPS in RAW264.7 cells through inhibition of NF-κB and MAPKs signaling" was published in 2020. Journal: Biosci Rep.

**Figure 2:** Effects of SOG on Raw264.7 macrophages’ viability Raw264.7 cells were treated with SOG (25, 50 and 100 μM) or DMSO (vehicle) for 24 h in the presence of 500 ng/ml LPS. Values are indicated relative to cells processed by the vehicle, which are normalized to 100%. The values of three independent experiments were expressed as mean ± SEM.

### Effect of SOG on mRNA expression of inflammatory mediators in mouse peritoneal macrophages activated by LPS

In order to determine the anti-inflammatory activity of SOG, the effect of SOG on the expression of mRNA for TNF-α and IL-6 in LPS stimulated mouse macrophages were further investigated. As shown in Figure 3, levels of TNF-α and IL-6 mRNA in LPS treated mouse macrophages attenuated in a dose-dependent manner of SOG. The results indicated that SOG inhibited the expression of TNF-α and IL-6 induced by LPS via blocking the transcription of these genes.

**Figure 3:** SOG reduced the mRNA levels of inflammatory mediators Indicated concentrations of SOG (25, 50 and 100 μM) were added to RAW 264.7 cells stimulated by LPS. RAW 264.7 cells were collected and RNA samples were prepared after incubating 6 h. The mRNA degrees of TNF-α (**A**) and IL-6 (**B**) were detected using RT-real time PCR. The results of three independent experiments were expressed as means ± SEM. *P < 0.05, **P < 0.01 and ***P < 0.001 versus group treated by LPS.

### Effects of SOG on NF-κB activation in RAW264.7 macrophages stimulated by LPS

NF-κB signaling pathways play an important role in the inflammatory response of macrophages to external stimulation. In resting macrophages, NF-κB is certainly bound to its inhibitor IκB, and confined to the cytoplasma. When stimulated by an external signal such as LPS, IκB is demerged, and NF-κB is released and transported to nucleus, promoting transcription of targeted genes including TNF-α and IL-6 [12,13]. To further address the underlying mechanism of inhibiting the gene expression of inflammatory cytokine by SOG, the effect of SOG on NF-κB activation induced by LPS is explored. As shown in Figure 4, LPS stimulation significantly enhanced the phosphorylation of NF-κB p65 subunit, and the degradation of IκB-α. IκB-α degradation and NF-κB p65 phosphorylation have been suppressed by SOG treatment.

**Figure 4:** The effects of SOG on NF-κB activation in RAW264.7 cells stimulated by LPS Indicated doses of SOG (25, 50 and 100 μM) or DMSO (vehicle) were added to cells 30 min before LPS stimulation. RAW264.7 cells were collected and protein samples were prepared after LPS treatment for 15 minutes. (**A**) The degradation of IκB-α and phosphorylation of NF-κB p65 subunit were assessed using Western blot assay. (**B**) Band density was measured using ImageJ software. The relative levels of target proteins were compared between samples. The results of three independent experiments were expressed as means ± SEM. ^#^*P* < 0.05, ^##^*P* < 0.01 and ^###^*P* < 0.001 versus group treated by vehicle; ***P < 0.001 versus group treated by LPS.

The article "Sec-O-glucosylhamaudol suppressed inflammatory reaction induced by LPS in RAW264.7 cells through inhibition of NF-κB and MAPKs signaling" was published in 2020. Journal: Biosci Rep.

### SOG reduced MAPK phosphorylation induced by LPS

Phosphorylation of MAPKs, including JNK, p38 and ERK1/2, activate transcription factor AP-1, and then transcribe inflammatory mediators [13,14]. To determine whether SOG suppressed inflammatory cytokine expression via modulation of MAPK signaling, the effects of SOG on phosphorylation of ERK1/2, JNK and p38 in macrophages induced by LPS were measured. As shown in Figure 5, SOG treatment suppressed LPS-induced MAPK phosphorylation. In conclusion, results suggested that SOG plays an anti-inflammatory role by blocking MAPK phosphorylation and NF-κB activation in macrophages stimulated by LPS.

**Figure 5:** The effects of SOG on p38, JNK as well as ERK1/2 Indicated doses of SOG (25, 50 and 100 μM) or DMSO (vehicle) were added to cells 30 min before LPS stimulation. Cells were collected and protein samples were prepared after LPS treatment for 15 minutes. (**A**) Total and phosphorylated MAPKs including JNK, p38 and ERK1/2 were evaluated using western blot assay. (**B**) ImageJ software was employed to quantify band density. The relative levels of target proteins were compared between samples. The results of three independent experiments were expressed as means ± SEM. ^##^*P* < 0.01 and ^###^*P* < 0.001 versus group treated by vehicle; ***P < 0.001 versus group treated by LPS.

## Discussion

As the first line of host defense, innate immunity system serves as a critical part in keeping tissue homeostasis and responding to external pathogenic stimuli or internal insults. Macrophages and neutrophils are the main effector cells of the innate immunity response. It was found that SOG could reduced the expression of inflammatory mediators including TNF-α and IL-6 via suppressing the MAPK phosphorylation and NF-κB activation in Raw264.7 murine macrophages induced by LPS.

Activated macrophages could produce and release pro-inflammatory cytokines, such as TNF-α, IL-6, NO and PGE2, which thus played a key role in inflammatory diseases such as sepsis, rheumatoid arthritis, inflammatory bowel disease, psoriasis and Type 2 diabetes [1,15]. SOG reduced the release and transcription of inflammatory cytokines including TNF-α and IL-6 in a dose-dependent manner. In short, these results suggested that SOG exert its anti-inflammatory effects via reducing inflammatory medium expression in LPS-stimulated macrophages. Several studies have shown that the pro-inflammatory cytokines, including TNF- α and IL-6, in macrophages stimulated by LPS were mainly dependent on NF-κB signaling pathway [1,17,18]. Activating NF-κB includes ubiquitination, phosphorylation and following IκB- α degradation by the 26S proteasome. NF-κB was released from the cytoplasmic NF-κB–IκB-α complex, and free NF-κB was translocated into the nucleus, in which it was bound to NF-κB sites in the promoter region of genes for some pro-inflammatory cytokines or inflammatory mediators [4,16]. Several previous studies reported that some natural compounds such as schisantherin A, sauchinone and arctigenin exerted their anti-inflammatory impact by blocking MAPK and NF-κB signaling pathways [19–21]. To investigate whether SOG can inhibit the expression of TNF-α and IL-6 in LPS-stimulated RAW264.7 cells via blocking NF-κB signaling pathway, the effects of SOG on the degradation of IκB-α degradation and NF-κB p65 subunit phosphorylation were thus measured. As demonstrated in Figure 4, LPS-induced IκB-α degradation and NF-κB p65 subunit phosphorylation were repressed by SOG treatment dose-dependently, indicating that SOG plays an anti-inflammatory role by regulating NF-κB signaling pathway.

The article "Sec-O-glucosylhamaudol suppressed inflammatory reaction induced by LPS in RAW264.7 cells through inhibition of NF-κB and MAPKs signaling" was published in 2020. Journal: Biosci Rep.

MAPK signaling pathway plays an important role in many biological procedures, such as inflammation, apoptosis and proliferation [4]. Several studies have shown that induced expression of iNOS, COX-2, TNF- α or IL-6 were controlled by activation of ERK1/2, p38 and JNK, which belong to MAPK family [4,22]. To explore whether MAPK pathway mediated by LPS is involved in the inhibition of SOG against inflammation induced by LPS, we examined the effect of SOG on MAPK phosphorylation. The results were shown in Figure 5, SOG treatment dose-dependently attenuated the phosphorylation of ERK1/2, p38 and JNK induced by LPS in the Raw264.7 macrophages. Taking together, SOG suppressed the expression of IL-6 and TNF-α in Raw264.7 macrophages stimulated by LPS through suppressing the activation of MAPK and NF-κB signaling pathway.

In conclusion, we report for the first time that SOG has anti-inflammatory activity in LPS-induced RAW264.7 macrophages and its possible anti-inflammatory mechanism. However, whether SOG could exert anti-inflammatory effect *in vivo* remains unclear and further *in vivo* study should be conducted using inflammatory disease animal model. Our research shows that SOG might provide effective and secure treatment choices for various disorders mediated by inflammation.

The article "Sec-O-glucosylhamaudol suppressed inflammatory reaction induced by LPS in RAW264.7 cells through inhibition of NF-κB and MAPKs signaling" was published in 2020. Journal: Biosci Rep.

## Abbreviations

DMSO: dimethyl sulfoxide
ELISA: enzyme-linked immunosorbent assay
FBS: fetal bovine serum
5-LOX: 5-lipoxygenase
MTT: 3-(4,5-dimethylthiazol-2-yl)-2,5-diphenyl tetra-zolium bromide
SOG: sec-O-glucosylhamaudol
